# Analysis of miRNA signature differentially expressed in exosomes from adriamycin-resistant and parental human breast cancer cells

**DOI:** 10.1042/BSR20181090

**Published:** 2018-11-16

**Authors:** Wei-xian Chen, Ling-yun Xu, Qi Qian, Xiao He, Wen-ting Peng, Yu-lan Zhu, Lin Cheng

**Affiliations:** Department of Breast Surgery, The Affiliated Changzhou No. 2 People’s Hospital of Nanjing Medical University, Changzhou, China

**Keywords:** Breast cancer, Chemoresistance, Exosomes, MicroRNA

## Abstract

A major cause of failure in chemotherapy is drug resistance of cancer cells. Exosomes have been introduced to spread chemoresistance through delivering miRNAs. However, a systematic evaluation of the exosomal miRNA expression profiles responsible for chemoresistance is still lacking. In the present study, miRNA signature differentially expressed in exosomes derived from adriamycin-resistant (A/exo) and parental breast cancer cells (S/exo) were analyzed by microarray and the results were confirmed by PCR. A total of 309 miRNAs were increased and 66 miRNAs were decreased significantly in A/exo compared with S/exo. Specifically, 52 novel miRNAs with increased expression levels >16.0-fold in A/exo were identified. After prediction of target genes for 13 of 52 selected novel miRNAs, pathway analysis, gene ontology (GO) terms, and protein–protein interactions (PPIs) were constructed. The results implied that these selected exosomal miRNAs inhibited target genes involved in transcriptional misregulation in cancer, MAPK, and Wnt signaling pathways. Functional enrichment analysis demonstrated that the target genes were mainly responsible for protein phosphorylation, transcription regulation, molecular binding, and kinase activity. In summary, the current bioinformatics study of exosomal miRNAs may offer a new understanding into mechanisms of chemoresistance, which is helpful to find potential exosomal miRNAs to overcome drug insensitivity in future breast cancer treatment.

## Introduction

Breast cancer is the most common malignant tumor resulting in high mortality amongst females worldwide [1]. Although chemotherapy plays an important role in breast cancer treatment, drug resistance, whether innate or acquired over time, minimizes the effectiveness of antineoplastic agents in a large number of patients and remains the major cause of clinical treatment failure [2]. Unresponsiveness of tumor cells to toxic insult is a complex phenomenon. To date, much attention has been paid to study the multiple factors and molecular machinery of chemoresistance; however, the underlying mechanisms are still poorly understood.

Exosomes are small vesicles of endocytic origin approximately 50–100 nm in diameter released by various cell types. Growing evidence revealed that exosomes are significant regulators in cancer biology, including tumorigenesis, angiogenesis, invasion, and metastasis [3]. Resistance transmission is also one such role, through their ability to travel within tumor microenvironment and shuttle a wide variety of active molecules including proteins, lipids, and especially miRNAs [4,5]. Xiao et al. [6] reported that exosomes and the contained *miR-21* and *miR-133b* were involved in the regulation of sensitivity of lung cancer cells to cisplatin exposure. Wei et al. [7] found that exosomes from tamoxifen-resistant breast cancer cells could enter into sensitive cells and release *miR-221/222*, leading to reduced target genes expression and enhanced drug resistance in recipient cells. Our recent work indicated that docetaxel-resistant breast cancer cells were able to spread chemoresistance to sensitive cells by releasing abundant exosomes and transferring specific miRNAs [8]. Accumulating research has, thus far, been conducted to support the hypothesis that exosomal miRNAs could be tied to respond to anticancer agents [5].

Given that most previous studies attempting to detect miRNA signature relevant to chemosensitivity and therapy resistance have scanned only cellular miRNAs or detected only individual exosomal miRNA, it is becoming necessary to assess the exosomal miRNA expression profiles. Therefore, the purpose of the present study was to comprehensively evaluate the miRNA signature differentially expressed in exosomes derived from adriamycin-resistant and parental breast cancer cells. Bioinformatics analysis was also performed to predict target genes of the dysregulated exosomal miRNAs and to understand their potential functions in the formation of chemoresistance.

## Materials and methods

### Cell culture

Human breast cancer cell line MCF-7 was obtained from the Cell Bank of the Chinese Academy of Sciences (Shanghai, China). The adriamycin-resistant variant of MCF-7 cells (MCF-7/Adr) was established from the parental sensitive cell line (MCF-7/S) by continuous culture in medium containing stepwise increasing concentrations of adriamycin in our laboratory as recently described [9]. All cell lines were incubated in Dulbecco’s modified Eagle’s medium (DMEM) high glucose (HyClone, U.S.A.) supplemented with 10% FBS, 100 U/ml penicillin, and 100 μg/ml streptomycin in an atmosphere of 5% CO_2_ at 37°C. Exosome-free FBS was prepared by ultracentrifugation (Avanti J-30I, Beckman Coulter, U.S.A.) at 100000***g*** and used for all studies.

### Exosome isolation and identification

Exosomes were isolated from medium of MCF-7/Adr and MCF-7/S using repeated centrifugation and ultracentrifugation steps and respectively named as A/exo and S/exo for simplicity. They were used immediately or resuspended in 1 ml PBS and stored at −80°C. Exosomes were subsequently characterized using the methods that we recently reported [8]. Briefly, 10 μl exosome samples were placed on parafilm and covered with a 300-mesh copper grid for 45 min. Then, the copper mesh was washed thrice by PBS, fixed in 3% glutaraldehyde for 10 min, washed thrice with double distilled water, and finally contrasted in 2% uranyl acetate. The shape and size of exosomes were examined using a JEM-1010 electron microscope (JEOL, Japan) at an accelerating voltage of 80 kV.

### Exosomal miRNA extraction and microarray

Exosomal RNA was extracted using the Total Exosome RNA and Protein Isolation Kit (Invitrogen, U.S.A.) in accordance with the manufacturer’s protocols. RNA was quantitated spectrophotometrically (Thermo Scientific, U.S.A.), and the integrity was assessed by an Agilent 2100 Bioanalyzer (Agilent Technologies, U.S.A.). Microarray hybridization and analysis were carried out as previously described, using Affymetrix GeneChip miRNA 3.0 Array, which contains 1733 human mature miRNA probe sets [10]. Differentially expressed miRNAs were filtered to exclude those changes less than 2.0-fold compared with S/exo.

### Real-time PCR

Total RNA including miRNA was stem-loop reverse transcribed to cDNA using the SYBR PrimeScript RT-PCR kit (Takara Bio Inc., Japan) on an iCycler iQ system (Bio-Rad, U.S.A.). Real-time PCR was conducted on a Light Cycler 480 (Roche, Australia) with the same kit according to the manufacturer’s protocols. All reactions, including the no-template controls, were performed in a 20-μl reaction volume in triplicate. The primers for *U6* are as follows: forward, 5′-CGCAAGGATGACACG-3′; reverse, 5′-GAGCAGGCTGGAGAA-3′. The relative miRNA expressions were calculated using ΔΔ*C*_t_ method and normalized to *U6*.

### Target genes prediction

Target genes of the selected miRNAs were predicted by starBase V2.0 (http://starbase.sysu.edu.cn/browseClipSeq.php) which is a database for exploring miRNA–mRNA interaction maps, combining five prediction programs (TargetScan, PicTar, RNA22, PITA, and miRanda) [11]. Since the prediction software often suffers from high false positive rates, only the genes listed by at least four independent tools were taken into account.

### Kyoto Encyclopedia of Genes and Genomes pathway analysis and gene ontology annotation

Kyoto Encyclopedia of Genes and Genomes (KEGG) pathway enrichment analysis and gene ontology (GO) analysis were performed using the DAVID program (http://david.abcc.ncifcrf.gov/) [12–14]. The count number larger than 2 and Bonferroni *P*-value <0.05 were chosen as the threshold. Cytoscape 3.1.1 (http://cytoscape.org/) was used to construct the possible functional network [15].

### Integration of protein–protein interaction network

Target genes of dysregulated miRNAs were uploaded to the Search Tool for the Retrieval of Interacting Genes (STRING) database (http://www.string-db.org/) to assess protein–protein interaction (PPI) information [16]. Combined score >0.4 was set as significant. The plug-in Molecular Complex Detection (MCODE) was used to select the modules of PPI network in Cytoscape software. Then, pathway enrichment analysis was performed for genes in the modules.

### Statistical analysis

Data were analyzed using the SPSS 20.0 package. All experiments were done in triplicate and the data presented were representative of three independent experiments. Statistical significance was assumed when *P*<0.05.

## Results

### Exosome characterization

To ensure successful isolation of exosomes from MCF-7/Adr and MCF-7/S cells, the collected A/exo and S/exo were observed by TEM. Exosomes exhibited spheroid shape measuring 50–100 nm in diameter (Figure 1A,B). A bioanalyzer profile of total RNA present in A/exo and S/exo showed that exosomal RNAs were small RNAs (Figure 1C,D).

**Figure 1:** Exosome characterization (**A**) Representative micrograph of TEM of A/exo (scale bar = 200 nm). (**B**) Representative micrograph of TEM of S/exo (scale bar = 200 nm). (**C**) A bioanalyzer profile of total RNA showed that A/exo were enriched in small RNAs. (**D**) A bioanalyzer profile of total RNA showed that S/exo were enriched in small RNAs.

### Expression profile of exosomal miRNAs

We carried out a microarray analysis of small RNAs in A/exo and S/exo and categorized them into miRNA, CDBox, HacaBox, scaRNA, and snoRNA according to the manufacturer’s instructions. Approximately 71% from A/exo and 52% from S/exo were mapped on to miRNAs (Figure 2A,B). Compared with miRNAs in S/exo, 309 miRNAs were up-regulated and 66 miRNAs were down-regulated significantly in A/exo (at least 2.0-fold changes). Amongst these differentially expressed miRNAs, A/exo had a total of 52 novel miRNAs with increased expression levels >16.0-fold and 4 novel miRNAs with reduced expression levels >16.0-fold of the corresponding miRNAs in S/exo (Table 1). Hierarchical cluster analysis revealed that A/exo and S/exo were characterized by significant changes in miRNA expression (Figure 2C).

**Figure 2:** Expression profile of exosomal miRNAs (**A**) Pie chart for small RNAs in A/exo. (**B**) Pie chart for small RNAs in S/exo. (**C**) Hierarchical cluster analysis of miRNA expression profiles in A/exo compared with S/exo. Black color stands for a median transcript level. Yellow and blue color stand for a transcript level above and below the median level, respectively. (**D**) The PCR results correlated well with the microarray data.

**Table 1:** The novel miRNAs with expression levels >16.0-fold in A/exo compared with S/exo

Up-regulated miRNAs	Log2 (fold change)*	Down-regulated miRNAs	Log2 (fold change)
hsa-let-7b-5p_st	5.23	hsa-miR-1263_st	−4.36
hsa-miR-1202_st	5.47	hsa-miR-3613-5p_st	−5.54
hsa-miR-1225-5p_st	4.47	hsa-miR-3927_st	−4.07
hsa-miR-1231_st	4.10	hsa-miR-455-3p_st	−4.87
hsa-miR-1246_st	6.00		
hsa-miR-1307_st	5.13		
hsa-miR-150-star_st	5.29		
hsa-miR-1587_st	5.47		
hsa-miR-16-5p_st	4.72		
hsa-miR-17-5p_st	4.62		
hsa-miR-181a-5p_st	4.71		
hsa-miR-1909_st	4.09		
hsa-miR-1910_st	4.48		
hsa-miR-191_st	5.18		
hsa-miR-193a-3p_st	6.43		
hsa-miR-193b-3p_st	4.67		
hsa-miR-194_st	6.45		
hsa-miR-2276_st	6.00		
hsa-miR-23a-3p_st	7.03		
hsa-miR-23b-3p_st	5.66		
hsa-miR-26a-5p_st	4.33		
hsa-miR-27a-3p_st	4.43		
hsa-miR-30a-5p_st	4.73		
hsa-miR-3135b_st	4.40		
hsa-miR-3164_st	4.54		
hsa-miR-3180-3p_st	4.27		
hsa-miR-3180_st	4.07		
hsa-miR-3188_st	5.06		
hsa-miR-3192_st	4.82		
hsa-miR-320a_st	4.22		
hsa-miR-328-3p_st	4.84		
hsa-miR-3652_st	4.15		
hsa-miR-3663-3p_st	6.23		
hsa-miR-3691-3p_st	4.38		
hsa-miR-3944-3p_st	4.26		
hsa-miR-4269_st	7.00		
hsa-miR-4271_st	4.44		
hsa-miR-4327_st	5.11		
hsa-miR-4461_st	4.78		
hsa-miR-4486_st	4.62		
hsa-miR-4539_st	4.50		
hsa-miR-4667-5p_st	5.34		
hsa-miR-4700-5p_st	5.14		
hsa-miR-4708-5p_st	4.99		
hsa-miR-4725-3p_st	4.96		
hsa-miR-4750_st	6.28		
hsa-miR-4767_st	4.82		
hsa-miR-4778-5p_st	4.78		
hsa-miR-4800-3p_st	4.54		
hsa-miR-483-5p_st	4.54		
hsa-miR-874_st	5.03		
hsa-miR-939_st	4.84		

* Fold change = (A/exo)/(S/exo).

We next selected five differentially expressed exosomal miRNAs, which could be found in starBase database, for PCR validation. These selected miRNAs covered both top up-expressed miRNAs (*miR-23a-3p, miR-27a-3p, miR-30a-5p*, and *miR-320a*) and top down-expressed miRNAs (*miR-455-3p*) in A/exo. In all cases, the PCR results correlated well with the microarray data (Figure 2D).

### Analysis of involved pathways

To understand which pathway might be involved in chemoresistance formation, we predicted the potential target genes of the most abundant miRNAs in A/exo. Based on prediction, a total of 13 exosomal miRNAs found in starBase database (*miR-16-5p, miR-17-5p, miR-23a-3p, miR-23b-3p, miR-26a-5p, miR-27a-3p, miR-30a-5p, miR-181a-5p, miR-193a-3p, miR-193b-3p, miR-320a, miR-328-3p*, and *let-7b-5p*) were expected to target 1762 genes. From the results, we found that a single miRNA could target hundreds of genes and a single gene could be targetted by multiple miRNAs. Then, predicted genes were assigned into KEGG pathway, and Cytoscape software was used to decipher the possible functional network. We discovered 24 pathways, of which the ‘transcriptional misregulation in cancer’ was the most prominent (Figure 3). Moreover, KEGG analysis offered us further information that ‘transcriptional misregulation in cancer’ was the important pathway that gathered most target genes of eight miRNAs, including *miR-17-5p* (14 genes), *miR-23a-3p* (7 genes), *miR-23b-3p* (8 genes), *miR-27a-3p* (8 genes), *miR-181a-5p* (7 genes), *miR-193a-3p* (4 genes), *miR-193b-3p* (4 genes), and *miR-328-3p* (3 genes). Several other significant pathways were also detected, e.g. ‘MAPK signaling pathway’, ‘Pathways in cancer’, and ‘Wnt signaling pathway’ (Figure 3). In breast cancer, these signaling pathways are generally associated with drug resistance and treatment failure [17,18].

**Figure 3:** Analysis of involved pathways KEGG pathway analysis of target genes of 13 most abundant miRNAs in A/exo showed a functional network. Red rhombus stands for exosomal miRNA. Blue ellipse stands for signaling pathway.

### Analysis of GO enrichment

To comprehensively explore the biological functions of target genes, we performed GO enrichment analysis, including biological process, molecular function, and cellular component. The analysis of biological process indicated that the selected miRNAs were mainly responsible for ‘positive/negative regulation of transcription from RNA polymerase II promoter’, ‘protein phosphorylation/dephosphorylation’, and ‘positive/negative regulation of transcription, DNA-templated’. Other categories such as ‘cell cycle’, ‘cell migration’, ‘apoptotic process’, and ‘cell proliferation’ were also enriched (Figure 4). The analysis of molecular function revealed that the selected miRNAs were associated with various functions, and most of them were related to ‘protein binding’, ‘DNA binding’, and ‘kinase activity’ (Figure 5). The analysis of cellular component showed that the selected miRNAs were involved in ‘nucleus’, ‘cytoplasm’, ‘nucleoplasm’, ‘cytosol’, and ‘membrane’ (Figure 6).

**Figure 4:** GO enrichment analysis of biological process of the target genes Red rhombus stands for exosomal miRNA. Blue ellipse stands for biological process.

**Figure 5:** GO enrichment analysis of molecular function of the target genes Red rhombus stands for exosomal miRNA. Blue ellipse stands for molecular function.

**Figure 6:** GO enrichment analysis of cellular component of the target genes Red rhombus stands for exosomal miRNA. Blue ellipse stands for cellular component.

### Analysis of PPI network

To evaluate PPI information, we mapped the target genes of the selected miRNAs to STRING database. According to the profile obtained from STRING tool, the PPI network consisted of 1569 nodes and 15449 edges. Given that PPI network contains numerous nodes and interactions, the top three highest modules was selected by using plug-in MCODE. Several hub genes including *CCND2, CXCL12*, and *PTEN* were identified. Enrichment pathway analysis showed that the genes in the modules were related to ‘Pathways in cancer’, ‘PI3K/Akt signaling pathway’, and ‘MAPK signaling pathway’ (Figure 7).

**Figure 7:** Analysis of PPI network (**A**) Module 1. (**B**) The enriched pathway of module 1. (**C**) Module 2. (**D**) The enriched pathway of module 2. (**E**) Module 3. (**F**) The enriched pathway of module 3.

## Discussion

The underlying mechanisms for drug resistance remain largely unexplored. Investigating the molecular machinery of chemoresistance has therefore become an emergent issue in breast cancer treatment [2]. Our recent studies, along with several other findings, have confirmed that exosomal miRNAs play an important role in the development of chemoresistance [7,8]. In the present work, we checked the miRNA expression profiles that were differentially expressed between A/exo and S/exo. We then performed function analysis for the predicted target genes of novel exosomal miRNAs with KEGG pathways, GO enrichment, and PPI network.

In all the miRNAs shared by both exosomes, 309 miRNAs were elevated and 66 miRNAs were reduced significantly in A/exo, indicating that the exosomes from adriamycin-resistant breast cancer cells were characterized by significant changes in miRNA expression. Amongst the 52 novel miRNAs overexpressed, *miR-23a-3p* was found to have the greatest expression fold-change between A/exo and S/exo. This miRNA has been previously reported to promote breast cancer cell invasion and hepatic metastasis [19]. The expressions of selected exosomal miRNAs were validated by PCR, and the results were correlated well with our microarray data.

In order to better understand the interactions of target genes in chemoresistance formation, KEGG analysis was performed to identify predominant pathways. The results showed that the predicted target genes of 13 specific exosomal miRNAs were enriched in 24 pathways, of which the ‘transcriptional misregulation in cancer’ was the most prominent. Several other classical pathways detected from the top enriched KEGG terms, namely MAPK, Wnt, PI3K/Akt, TGF-β, and Hippo signaling pathways, have been previously confirmed to be responsible for drug resistance [17,18,20,21]. The ‘axon guidance’ is important not only in tumorigenesis and tumor progression, but also in breast cancer therapy [22]. Since cancer stem cells are a subpopulation of malignant cells with self-renewal capability that contribute to tumor propagation and metastasis, studying the genes in ‘signaling pathways regulating the pluripotency of stem cells’ would also help us to uncover mechanisms of chemoresistance [23]. Further investigations are needed to more precisely elucidate the relevance of these signaling pathways.

Functional enrichment analysis demonstrated that the target genes of exosomal miRNAs were mainly involved in protein phosphorylation, transcription regulation, molecular binding, and kinase activity. This is consistent with the knowledge that defects of biological process, molecular function, and cellular component are main causes for tumor development and progression [24]. It is desired that further attention be drawn to this field. PPI network may aid in uncovering the potential mechanism of chemoresistance; however, it contains numerous nodes and interactions, which is difficult to draw the useful information for us. Therefore, the top three highest modules were constructed and several hub genes were identified. CCND2 forms a complex with CDK4 and functions as a regulatory subunit of the complex, whose activity is required for cell cycle G_1_/S transition [25]. CXCL12 modulates cell proliferation, apoptosis, migration, and angiogenesis in various cancers including breast cancer. Drug design targetting CXCL12 pathway is well reviewed as a promising anticancer strategy [26]. *PTEN*, one of the most altered tumor suppressor genes which functions to antagonize the PI3K activity and inhibit cell proliferation, was reported to regulate multidrug resistance of breast cancer [10,27]. Our previous studies have also confirmed that miRNAs delivered by exosomes were able to suppress PTEN expression [8]. Further analysis showed that the genes in the modules were mainly related to ‘Pathways in cancer’, ‘PI3K/Akt signaling pathway’, and ‘MAPK signaling pathway’. As a matter of fact, these signaling pathways are generally associated with drug resistance and treatment failure in breast cancer [17,27]. Although the current study is a bioinformatics analysis, we still believe that miRNAs packaged in A/exo can be delivered into recipient cells and act as physiologically functional molecules to exert gene silencing through the same mechanism as endogenous miRNAs. These appear likely because our previous group have demonstrated that exosomal *miR-1246*, a novel miRNA in Table 1, could suppress Cyclin-G2 and promote cell proliferation, invasion pathways, and drug resistance in breast cancer [28].

In conclusion, the present work provides a comprehensive bioinformatics analysis of the miRNA signature differentially expressed in exosomes derived from adriamycin-resistant and parental breast cancer cells. KEGG pathways, GO terms, and PPI network of 13 most abundant miRNAs in A/exo were analyzed to understand their potential functions in the development of chemoresistance. Remarkably, the study of linking different exosomal miRNAs to various target genes and pathways is still in infancy stage. Further experimental excavation and research are needed to investigate the functionally relevant target genes and pathways of exosomal miRNAs in chemoresistance formation.

## Abbreviations

GO: gene ontology
KEGG: Kyoto Encyclopedia of Genes and Genomes
MCODE: Molecular Complex Detection
PPI: protein–protein interaction
STRING: Search Tool for the Retrieval of Interacting Genes
